The article "Green Supply Chain Management and Its Impact on Economic-Environmental Performance: Evidence from Asian Countries" was retracted in 2023. Reasons: unreliable results or conclusions; concerns about the data; concerns about the peer review; concerns about the citations.

# Green Supply Chain Management and Its Impact on Economic-Environmental Performance: Evidence from Asian Countries

**DOI:** 10.1155/2022/7035260

**Published:** 2022-09-20

**Authors:** Huihua Huang

**Affiliations:** Economic and Trade College, Hunan Vocational College of Commerce, Hunan, China

## Abstract

At present, with the increasing seriousness of ecological pollution, people are gradually paying more attention to the protection of the ecological environment. In the past, people only paid attention to economic growth and neglected environmental protection. Now, environmental problems have restricted economic development, leading scholars at home and abroad to reflect on it deeply. Supply chain management, as the key to the sustainable development of the current enterprise economy, can realize the key consideration of environmental factors in the complete supply chain, reduce the negative impact of economic production activities on environmental protection, and can also make better use of resources to achieve effective assessment of the impact of economic-environmental performance in the supply chain process to ensure its healthy and orderly development. This article makes an in-depth analysis of the use of a green supply chain in the impact of economic-environmental performance by using the method of a fuzzy comprehensive evaluation and provides a relatively complete calculation method. An example is given to analyze the IKEA company. The results of the example analysis show that green supply chain management not only promotes economic growth in economic-environmental performance but also plays a continuous role in the improvement of the environment. The proportion of resource consumption in regions with a high level of economic development is also high. Driven by factors of green supply chain management, green economy can effectively alleviate environmental pollution and further promote economic and green sustainable development.

## 1. Introduction

In essence, the supply chain is to use the orderly combination of raw material suppliers, product manufacturers and processors, commodity marketers, and purchasing customers to form a chain system. Supply chain management can effectively meet basic needs and effectively combine the basis of each supply chain node. The traditional cargo supply chain management can take the maximization of the utilization of the entire supply chain system as the development goal and can fully consider the content of noneconomic factors, such as the impact on society and the environment. Research scholars from China and other countries have also carried out in-depth research on green supply chain management. Zhang Juan used a fuzzy judgment algorithm to study the entire performance evaluation model of the green supply chain; Zhang Li used a neural network algorithm to study the basic theory of the green supply chain; Bai Shizhen mainly built a green supply chain performance evaluation system from three dimensions of economic development, social stability, and environmental protection and combined the gray evaluation model to evaluate the performance of the green supply chain [1–3]. With the society's continuous emphasis on the sustainable development of environmental protection, foreign scholars have also carried out in-depth analysis on the development of the green economy. The results of Magat's research show that the green supply chain can be used to effectively solve the problem of environmental pollution, can also effectively promote the sustainable growth of the economy, and effectively solve the problem of mutual restriction between economic development and environmental pollution. The results of Rennings' research can be seen that in addition to typical spillover effects, green supply chains can also effectively reduce the effects of production or products on the external environment, that is, “double external effects”. As an effective means to solve environmental protection and sustainable economic development, green supply chain management in Asian countries is helpful in maintaining a competitive advantage in the process of economic integration. However, not all countries that can effectively implement green supply chain management can always maintain an absolute advantage in the process of sustainable economic development. Therefore, sustainable economic development constituted by green supply chain management plays a very important role. Green supply chain management, as a process that can effectively promote green and sustainable development in Asian countries, is mainly because green supply chain management has a certain role in promoting the sustainable economic development of emerging BRICS countries. According to the theory of sustainable economic development, the economic-environmental performance development can be regarded as a coordinated mode that affects national environmental protection and sustainable economic development [4–7]. In order to promote the continuous growth of the economy, in recent years, the economic development model in Asian countries has gradually led to the continuous deterioration of the environment and the rapid consumption of resources. According to the existing natural resource basis analysis, the continuous deterioration of the environment will play a restrictive role in the sustainable development of the economy of Asian countries. In order to effectively solve the environmental issues, the potential environmental threats can be turned into competitive advantages for sustainable development. Green supply chain management can avoid inefficiencies and fully improve the utilization of resources so that Asian countries can build and maintain new opportunities provided by the competitive process. However, because the process of green supply chain management requires continuous investment of capital and labor costs, in the process of traditional economic-environmental performance development and evolution analysis of green economy development [8, 9], the analysis of the development and evolution of economic-environmental performance is usually carried out. However, the two-dimensional map can only describe the relative height of the environmental plane information but cannot provide relatively complete economic data information. The current requirement of economic-environmental performance development requires a one-stop service system, which can provide strong support for life and allow the entire economic-environmental performance development to obtain the highest economic benefits, which is the overall goal of economic-environmental performance development in China. References [10–12]. The development of green economy has gradually become an important research direction for the sustainable development of the Chinese economy. Through an in-depth analysis of typical green economic development models in China and other countries, the commonality and characteristics of its development process are explored, and the regularity and innovation of the development process of building a green economy are effectively summarized.

The continuous development of the economy has made environmental pollution more and more serious, and China has begun to use green supply chain management to solve the problems in the process of economic-environmental development. By comparing the existing use of economic-environmental development, this article constructs an economic-environmental performance model and uses it to conduct an in-depth analysis of green economic development in Asian countries. It can be concluded that green supply chain management plays a role in promoting economic growth in Asian countries. Period differences in the utilization process of economic-environmental performance are described, and period comparisons are made. Finally, through the analysis of examples, the results show that the use of green supply chain management in Asian countries is analyzed, and the elastic characteristics of economic-environmental performance in Asian countries are revealed.

## 2. Evaluation Indicators in Green Supply Chain

In order to effectively improve economic-environmental performance development, it is necessary to conduct a real-time analysis of the goals in the development of the green economy. At the same time, it will bring more long-term benefits to various regions. By constructing a model, it evaluates the influencing factors between the development influencing factors and the environmental sustainability of each regional economy. The economic-environmental performance can be improved rapidly, and it can also promote the effective utilization of the green economy in various regions of the country. By comparing other development models, the path suitable for the development of the regional green economy is explored to provide solutions and a theoretical basis for the development of economic-environmental performance in Asian countries. By analyzing the relationship between green supply chain management and economic-environmental performance, this article innovatively links the two key internal resources of green development identification, green innovation concept, economic-environmental performance, and green innovation, the starting key steps from green supply chain management to building economic-environmental performance, and further improves the in-depth research on green entrepreneurship [13, 14].

As can be seen from Figure 1, the impact of environmental protection on enterprises and the positive effect of environmental supply chain management on green innovation technology are reflected in support of government policies. The effective implementation of environmental supply chain management is to effectively add incentive policies to the process of economic development costs under the premise of ensuring the maximization of economic benefits; costs can be incorporated into the process of environmental protection. Such changes will lead to changes in the equilibrium price and the relationship between output and price, and changes in the equilibrium price will cause changes in the equilibrium output. The benefits caused by green innovation technologies are mainly determined by changes in profits and green manufacturing efficiency.

In the process of green supply chain management, the economic development strategy and the process of environmental protection are guided by the development of economic-environmental performance, and green supply chain management is roughly divided into three dimensions: innovation, initiative, and potential hidden dangers. The market economy of Asian countries is constantly adjusting the commercial development opportunities between themselves and environmental protection. Green supply chain management is a strategic decision-making model for the coordinated development of the economy and environment in the field of green economy. Based on the effective combination of economic development principles and models, this article explores the potential laws of green economic development. Local governments and social groups in Asian countries are key stakeholders in economic-environmental performance, and their main goals and decisions will directly promote the development of green economy.

This article mainly determines and applies the corresponding indicators of green supply chain from multiple aspects, such as relevant indicators determination rules, preliminary selection of evaluation indicators, and optimization of selected indicators. Indicators are characteristic concepts that can reflect social or natural phenomena to some extent and perhaps specific data, the effective combination of relevant indicators to form an indicator system, to analyze relatively complex problems, and finally obtain relevant characteristics and changing laws. In the system of determining green supply chain evaluation indicators, it is necessary to follow the principles of comprehensiveness of evaluation and scientific and systematic selection of indicators and the formed indicator system should also be hierarchical. The relevant indicators are evaluated, and the relevant rules are determined and combined with indicators to better evaluate the green supply chain. The relevant indicators selected mainly include 14 financial indicators, 16 operational indicators, and 15 environmental protection indicators. Effectively combining the above indicators can better effectively evaluate the relationship between the input and output of the green supply chain and then comprehensively evaluate the overall performance of the green supply chain.

## 3. Research Methods and Data Sources

### 3.1. Research Method

The fuzzy comprehensive evaluation method mainly uses a relatively complete evaluation index system for events with multiple attributes to conduct a more comprehensive overall evaluation of the target. The fuzzy comprehensive evaluation algorithm used is mainly an analytical method to solve inaccurate information and incomplete problem description. Among many evaluation methods, fuzzy comprehensive evaluation can usually effectively analyze the relevant fuzzy factors. Therefore, the comprehensive evaluation of economic-environmental performance using the fuzzy comprehensive evaluation method is a very effective method. The distinguishing feature is that it can be used for evaluation to a certain extent based on the subjective thoughts of the evaluator.

### 3.2. Overall Performance Evaluation Model

Combined with the environmental performance evaluation results in the constructed evaluation index system, the index codes shown in Table 1 can be obtained according to the relevant research results or relevant regulations.

Build an economic-environmental performance evaluation index system. On the basis of the constructed index evaluation system, the set value of the first-level evaluation index is *A* = {*A*l, *A*2, *A*3, *A*4}, and each index corresponding to the constructed first-level index *A*_*i*_(*i*=1,2,3,4) contains N multiple secondary indexes. It can be expressed as *A*_*i*_={*A*_*i*1_, *A*_*i*2_, *A*_*i*3_,…, *A*_*iN*_}, in turn, and can be converted into the matrix form corresponding to the index system as follows:

(1) $$\begin{array}{c} A=\left[\begin{array}{c} \begin{array}{cccccc} A11 & A12 & A13 & A14 & A15 & A16 \end{array}\\ \begin{array}{ccc} A21 & A22 & A23 \end{array}\\ \begin{array}{ccc} A31 & A32 & A33 \end{array}\\ \begin{array}{cc} A41 & A42 \end{array} \end{array}\right]. \end{array}$$

Construct a matrix of relevant weight coefficients. According to the relevant weight evaluation rules, the weight value needs to be determined for any subindex, and the expression is as follows [15, 16]:

(2) $$\begin{array}{c} W=\left[\begin{array}{c} \begin{array}{cccccc} W11 & W12 & W13 & W14 & W15 & W16 \end{array}\\ \begin{array}{ccc} W21 & W22 & W23 \end{array}\\ \begin{array}{ccc} W31 & W32 & W33 \end{array}\\ \begin{array}{cc} W41 & W42 \end{array} \end{array}\right]. \end{array}$$

A fuzzy comprehensive evaluation is a relatively complex process, and its analysis and calculation process are mainly divided into the following:

The final calculated score of each similar level indicator is calculated as follows:

(3) $$\begin{array}{c} H_{in}=\sum_{i=1,j=1}^{Gi}X_{ij}. \end{array}$$

According to expression, *n* is expressed as the n-th index in the analysis database, Gi is the number of indexes with the equivalent level, and *X*_*ij*_ is the comparison score when the *i*-th index is compared with the *j*-th index.

Combined with the last evaluation value of each row of indicators, the average evaluation value of the corresponding indicators is calculated in turn, and the expression is as follows:

(4) $$\begin{array}{c} V_{i}=\sum_{n=1}^{N}\frac{H_{in}}{N}. \end{array}$$

According to expression (4), N represents the number of samples collected.

For the average estimated value of each indicator at the same level, the weight value of the corresponding indicator value can be calculated, and the expression is as follows:

(5) $$\begin{array}{c} W_{i}=\frac{V_{i}}{\sum_{i=1}^{Gi}V_{i}}. \end{array}$$

Combined with the operation value of each index, the evaluation index value can be determined according to the operation value, and the evaluation results of the management indicators in the green supply chain are divided into five grades: excellent, good, medium, qualified, and poor, corresponding to 100%, 80%, 60%, 40%, and 20% of the hundred-mark system, The evaluation matrix used is the evaluation fuzzy mapping corresponding to each evaluation factor in the project matrix, which can be divided into fuzzy ratings of a single factor and evaluation results of multiple related factors [17, 18].

For the kth factor *A*_*k*_ corresponding to a single evaluation factor, the relevant factor evaluation is performed. Then, for the evaluation of the j-th factor, the *S*_*j*_ relevant membership degree is represented by *R*_*ij*_ , and the correlation evaluation matrix formed according to the evaluation of a single factor needs to combine the subordinate factors *A*_*i*_ to the fuzzy matrix *R*_*i*_ of the relevant single factor.

For example, for each factor in the evaluation factor in *A*_*k*_, the related membership degree matrix relationship is expressed as follows:

(6) $$\begin{array}{c} A_{k}=K\left[\begin{array}{ccc} A_{k11} & A_{k12} & A_{k13}\\ A_{k21} & A_{k22} & A_{k23}\\ \cdots & \cdots & \cdots \\ A_{kg1} & A_{kg2} & A_{kg3} \end{array}\right]. \end{array}$$

In matrix, *A*_*kij*_ denotes that in the i-th related evaluation factor in *A*_*k*_ corresponding to the *j*-th related subordination relationship, there are g-related evaluation factors in *A*_*i*_ in total, and there are *t*-related contents in the related evaluation matrix.

According to the membership function used, the most important thing is to determine the function expression that can be used, and the relevant results can be obtained using the relevant fuzzy evaluation method [19–22]. Because there is a mutual relationship between different factors in the evaluation of green performance in the green supply chain; that is, each evaluation factor has a certain fuzzy correlation, and it can be concluded that there is no significant boundary between each evaluation factor, which will lead to its membership calculation not being able to calculate the quantitative factor membership evaluation method. The weight value calculated according to the evaluated relevant matrix can be fuzzy-transformed, and the obtained fuzzy evaluation matrix expression is as follows:

(7) $$\begin{array}{c} Y_{k}=W_{k}\cdot R_{k},\\ =\left\{Y_{k1},Y_{k2},\ldots ,Y_{kg}\right\}. \end{array}$$

The fuzzy comprehensive evaluation method mainly uses a single factor comprehensively to form a high-level evaluation matrix. The calculation process of a single evaluation factor is used to multiply *R*_*i*_ with the corresponding weight coefficient, a single evaluation factor can be obtained, and then the performance analysis result *Y*_*i*_ can be calculated.

Because the evaluation results of a single factor can utilize the high-level correlation matrix, the performance analysis results can be quickly calculated. The calculation method constantly needs the influence of all relevant factors and can also save evaluation information at different levels and finally use expressions *M*=*Y* · *S*^*T*^ for comprehensive relevant evaluations. *M* in the expression represents the performance analysis score; Y represents the matrix relationship corresponding to the performance analysis; *S*^*T*^ represents the score relationships at different levels in the analysis.

The manufacturing enterprises and professional recycling enterprises selected in this article all operate normally at this scale, and the unit output between the original materials and the scrapped materials can be effectively calculated. The launch of each unit of product is the construction scale, and each waste is ensured to be optimally processed. After meeting the data and information on market recycling, each unit of waste is processed, and the conversion rate of each link becomes 100% [23, 24]. Then the market demand function is expressed as *D*=*Q* − *αP*_1_^1^,  *α* > 0; among them, *Q* represents the product market capacity and *P*_1_^1^ represents the unit product sales price; the waste recycling expression is *V*=*g*+*μP*_2_,  *μ* > 0, P2 represents the unit waste recycling price, and g represents the amount of the waste that the consumer voluntarily returns when the waste recycling price of the unit is 0.

Combined with the “double externalities” of the green supply chain, the government needs to take the necessary reward and punishment methods for incentives. The excess part will not be rewarded; otherwise, the punishment will be executed. The reward and punishment function are expressed as *L*_3_=*θ*_3_(*η* − *η*_0_)*D*_3_: *θ*3 represents the reward and punishment factor in the unit product, *θ*3 > 0; when *η* > *η*0, *L*3 represents reward; when *η*<*η*0, L3 represents punishment. *i* is used to represent the reward and punishment method, *i* = 1,2,3, *L*_*i*_ represents the government's reward and punishment when the government adopts method *i*, *P*_1*i*_^1^ represents the unit product sales price, *P*_1*i*_^2^ represents the unit waste raw material purchase price, *P*_2*i*_ represents the unit waste recycling price, *V*_*i*_ represents the green output, *D*_*i*_ represents the total output, and *S*_1*i*_, *S*_2*i*_, and *S*_*Ti*_ represent the profits of manufacturing enterprises, professional recycling and processing enterprises, and integrated supply chains, respectively, so we can get the following:

Profit of manufacturing company:

(8) $$\begin{array}{c} S_{1i}=\left(P_{1i}^{1}-p-c_{1}^{m}\right)\left(1-\eta \right)D_{i}+\left(P_{1i}^{1}-P_{1i}^{2}-c_{i}^{r}\right)V_{i}+L_{i}. \end{array}$$

Profits from recycling:

(9) $$\begin{array}{c} S_{2i}=\left(P_{1i}^{2}-P_{2i}-c_{2}\right)V_{i}. \end{array}$$

Profit from supply chain:

(10) $$\begin{array}{c} S_{Ti}=\left(P_{1i}^{1}-p-c_{1}^{m}\right)D_{i}+\left(p+c_{1}^{m}-c_{1}^{r}-c_{3}-P_{3i}\right)V_{i}+L_{i}. \end{array}$$

In the process of implementing green supply chain management, companies of Asian countries can maintain certain advantages in the ever-changing international market. However, an in-depth research is needed on which model can effectively promote green development and green innovation. For the analysis of a single individual country, there is no comprehensive study of the differences in time. China is an economy in a new situation at present, and its development is of great significance. This article calls the profit change caused by the green supply chain as its green supply chain benefit. The higher the income of the green supply chain, the stronger the green supply chain power, and vice versa. The evaluation of the economic-environmental performance in the green supply chain calculated in this article comprehensively reflects the improvement of the economic-environmental performance after the enterprise implements the green supply chain system.

## 4. Empirical Analysis

Economic-environmental performance is a current unique economic development strategy that can maintain advantages within a certain range and can be viewed from three dimensions: economy, environment, and society. According to the analysis of the basic concept of environmental protection, the main advantage of competition among Asian countries is that it can effectively promote the sustainable development of the environment and bring competitive advantages to its sustainable development. The development of green economy can realize economic adjustment in Asian countries and enhance the coordination of green supply chain management by acting on economic scale, economic efficiency, and economic structure of Asian countries. First, in terms of economic scale adjustment, it can attract a large number of private capital and social capital into the green economy market, expand financing channels in Asian countries, and increase cash holdings in Asian countries. It can alleviate the problem of insufficient economic-environmental performance in Asian countries, especially in technology-based environmental protection. According to the research results, we can see the relationship between the growth of emerging economies and environmental sustainability [25, 26]. With the continuous increase of GDP per capita of Asian countries, the degree of environmental sustainability also experienced first a decrease, then an increase, and finally a downward trend. The economic analysis model constructed by Chinese experts conducts an in-depth analysis of the evaluation of relevant economic development factors, evaluates the factors affecting the development of the Chinese economy and the influencing factors of environmental sustainability, and obtains the accuracy of the economy-environment. This accuracy can be rapidly improved and can also facilitate efficient use of economic resources. In the environment of green supply chain management, while quickly adjusting the economic structure of Asian countries, it can provide an auxiliary role for environmental protection. This article takes the economic-environmental performance of IKEA's green supply chain as an example and uses the fuzzy performance analysis method to conduct related research.

In the research of IKEA about green supply channels, a brief summary of the environment of this supply channel was taken. First, the environmental protection-related staff of IKEA and the staff of the national environmental protection unit, along with invited relevant experts, form a professional team to conduct detailed research and evaluation of the environment of IKEA's green supply channels. Through detailed reports and indicators, a professional questionnaire was drawn. The professional team conducted on-the-spot investigations on IKEA's internal production lines, material suppliers, retail stores, and even the delivery of goods and scored and evaluated them. Finally, through the evaluation data of the professional team, it is reclassified, evaluated, and analyzed.

Through professional team scoring data, summarized data relationship chart is as follows:

(11) $$\begin{array}{c} R_{1}=\left\{\begin{array}{ccccc} 0.35 & 0.25 & 0.20 & 0.10 & 0.10\\ 0.55 & 0.35 & 0.10 & 0 & 0\\ 0.50 & 0.30 & 0.13 & 0.06 & 0.01\\ 0.29 & 0.26 & 0.19 & 0.16 & 0.10\\ 0.39 & 0.34 & 0.21 & 0.06 & 0\\ 0.42 & 0.31 & 0.16 & 0.05 & 0.06 \end{array}\right\},\\ R_{2}=\left\{\begin{array}{ccccc} 0.39 & 0.31 & 0.19 & 0.06 & 0.05\\ 0.51 & 0.34 & 0.10 & 0.04 & 0.01\\ 0.29 & 0.36 & 0.21 & 0.09 & 0.05 \end{array}\right\},\\ R_{3}=\left\{\begin{array}{ccccc} 0.45 & 0.39 & 0.10 & 0.04 & 0.01\\ 0.34 & 0.41 & 0.21 & 0.06 & 0\\ 0.32 & 0.33 & 0.14 & 0.14 & 0.07 \end{array}\right\},\\ R_{4}=\left\{\begin{array}{ccccc} 0.44 & 0.31 & 0.15 & 0.09 & 0.01\\ 0.33 & 0.42 & 0.15 & 0.05 & 0.05 \end{array}\right\}. \end{array}$$

The first step is to analyze the primary data through the method of weight calculation through a score of the professional personnel.

(12) $$\begin{array}{c} W=\left\{\begin{array}{cccc} 0.36 & 0.29 & 0.21 & 0.14 \end{array}\right\}. \end{array}$$

The above conclusions are drawn from the first score, in which the environment plays the largest role, the second utilization of energy, and then the economic benefits of development, and the data on sustainable development has the least relative impact. This set of data can prove that professional teams are particularly interested in the role of goods supply channels in the environment. From another perspective, it can be seen that the awareness of environmental protection is becoming more and more important in the hearts of citizens. Secondly, the utilization rate of energy also occupies a large position. Energy cannot be regenerated, and its significance to economic development is obvious to all. At the same time, we are also concerned about the loss of energy because the loss of energy plays an intuitive and important role in the supply channel of green goods [27, 28]. Materials and resources are reused to maximize the utilization rate. Because resources are nonrenewable, the reuse of resources is the trend of the situation, and the value of waste resources also needs to be paid attention to by people. In the case of important scores, the share of sustainable economic development, which occupies 14%, is the smallest.

The secondary indicator of green supply channel score is calculated by weight:

(13) $$\begin{array}{c} W_{1}=\left\{\begin{array}{cccccc} 0.10 & 0.24 & 0.21 & 0.16 & 0.09 & 0.20 \end{array}\right\}. \end{array}$$

*W *_1_ is the relevant weight in the important score, among which the largest weight is the situation of toxic substances, wastewater discharge, and garbage; these three indicators are higher than the other three quantities. The toxicity of garbage directly affects the environmental pollution in the region, affects the pollution of the ecological environment, and directly affects people's lives, which really leads to the destruction of the ecological environment. In addition, the issue of wastewater discharge directly affects the situation of water resources. The current industrial wastewater discharge will contain heavy metals and even directly affect the water resources of people's living environment. If there are no restrictions on the discharge of wastewater from each factory, it will directly affect the water quality of people's lives. China's current water quality problem has become the top priority of the government. Because this problem has not been solved in time, people have suffered from serious diseases and even serious deaths due to water pollution. Therefore, the treatment of this wastewater discharge problem is an important task; therefore, garbage disposal accounts for a large proportion in the first-level evaluation.

(14) $$\begin{array}{c} W_{2}=\left\{\begin{array}{ccc} 0.25 & 0.45 & 0.30 \end{array}\right\}. \end{array}$$

W2 represents the relevant weight value of the second-level index in the energy utilization under the first-level index. It can be concluded that the proportion of material usage is relatively large, which can be as high as 45%. Because the resource consumption used by the existing industrial development will become larger, it will also cause the excessive use of other nonrenewable resources on the earth and cause serious environmental degradation. For example, when the number of views is relatively simple, large-scale soil and water loss in forests will experience the amount of energy consumption from time to time, which will cause adverse environmental impacts. The resources used are also divided into nonrenewable energy and renewable energy.

(15) $$\begin{array}{c} W_{3}=\left\{\begin{array}{ccc} 0.42 & 0.29 & 0.29 \end{array}\right\}. \end{array}$$

W3 represents the relevant weight of the second-level indicator in the first-level indicator economic development degree, and the utilization rate of recyclable and old materials has the largest weight, accounting for 42%. The reuse of recyclable materials can give full play to its use value. Therefore, the reuse of recycled materials in green supply chain management should be considered.

(16) $$\begin{array}{c} W_{4}=\left\{\begin{array}{cc} 0.62 & 0.38 \end{array}\right\}. \end{array}$$

*W *_4_ is the relative weight of the secondary indicators in the primary indicator of economic sustainability, of which ecological efficiency accounts for 62%.

Based on *Y*_*k*_=*W*_*k*_ · *R*_*k*_(*k*=1,2,3,4), the following can be obtained:

Y 1= (0.449,0.304,0.154,0.059,0.035).
Y 2= (0.416,0.337,0.154,0.066,0.028).
Y 3= (0.376,0.384,0.146,0.079,0.015).
Y 4= (0.409,0.341,0.150,0.079,0.021).

Finally, the total membership correlation matrix is obtained through the corresponding calculation:

(17) $$\begin{array}{c} R=\left\{\begin{array}{ccccc} 0.449 & 0.304 & 0.154 & 0.059 & 0.035\\ 0.414 & 0.339 & 0.154 & 0.066 & 0.028\\ 0.376 & 0.384 & 0.144 & 0.081 & 0.015\\ 0.411 & 0.341 & 0.148 & 0.078 & 0.022 \end{array}\right\}. \end{array}$$

According to the weight coefficient $W=\left\{\begin{array}{cccc} 0.36 & 0.29 & 0.21 & 0.14 \end{array}\right\}$, the evaluation matrix *Y* =*W*·*R* = (0.419, 0.335, 0.154, 0.069, 0.025) of environmental performance management in the total green supply chain is calculated, and finally, the comprehensive score of economic-environmental performance in the green supply chain is calculated. *M*=*Y* · *S*^*T*^=81.12; the basic rating is good.

If the environmental supervision and management department manages according to low standards, then the foreign investment environment will have little impact on the environment; if the management of the environmental supervision and management department is conducted in compliance with low and moderate standards, then the quality of foreign investment will improve the environment, because the management of the current region has been improved, some industries with a poor economy and high pollution will migrate or withdraw from the market due to the cost of environmental treatment and the high cost of improving environmental treatment. Strong regulatory authorities should use strict management methods to play a decisive role in the governance of the market and the environment and ultimately promote the “green” upgrade of the industrial structure. At the same time, in order to reduce pollutant emissions, foreign-funded enterprises must increase the cost of environmental governance, thereby encouraging them to strengthen green technology innovation, promoting the improvement of regional environmental efficiency in the long run, and making up for the cost caused by government environmental regulation. On the other hand, many multinational companies are born out of developed countries with strict environmental supervision and prefer to adapt to strict environmental standards through green technology research and development; the foreign companies can gain a local competitive advantage in environmental technology. Therefore, a moderate increase in the level of environmental regulation is conducive to attracting the inflow of green FDI(Table 2).

## 5. Conclusion

The continuous development of the modern economy has put forward higher requirements for enterprises. Sustainable economic-environmental development will aggravate the shortage of resources and environmental pollution continuously, which also brings serious challenges to the development of enterprises. This article constructs an economic-environmental performance evaluation system by using the green supply management method and uses the fuzzy performance analysis method to analyze it in depth. On the basis of the existing economic-environmental performance impact assessment research results, the factors of green supply chain management are comprehensively considered, an economic-environmental performance impact assessment system is constructed, and the fuzzy performance analysis algorithm is applied to the economic-environmental performance impact assessment. This method effectively ensures the authenticity of the evaluation results of the economic-environmental performance impact assessment and plays a very important role in the economic-environmental performance in the green supply chain. It can provide a reliable theoretical basis for enterprises to effectively implement green supply chain management. The results of the case analysis show that compared with the traditional economic development model, it greatly reduces the aggravation of environmental sustainability, has a positive role in promoting the long-term development of the Chinese economy optimization, and also realizes the optimization of the Chinese economic structure.

## Figures and Tables

**Figure 1:** Structure of the impact of environmental protection on enterprises.

**Table 1:** Optimal Evaluation index coding.

Target	First-level indicator	Secondary indicators
Economic-environmental performance A	Environmental impact degree A1	Garbage ratio A11
		Toxic substance A12
		Effluent discharge A13
		CO_2_ emissions A14
		Other waste discharge A15
		Garbage disposal A16
	Energy usage A2	Energy use A21
		Material consumption A22
		Energy saving A23
	Economic development degree A3	Utilization rate of reusable old materials A31
		Product recovery rate A32
		Other material recycling A33
	Economic sustainability A4	Eco-efficiency A41
		Green economy A42

**Table 2:** Regression results of the panel threshold model.

Threshold variable	Corrected environmental pollution cases		Proportion of pollution control operating costs by industry	
	FDI scale indicator model 1	FDI quality indicator model 2	FDI scale indicator model 3	FDI quality indicator model 4
fdi_1	0.065^∗∗∗^	0.028	0.052^∗^	−0.034
	(3.77)	(1.38)	(1.84)	(−1.43)
fdi_2	0.042^∗∗^	−0.024^∗∗^	0.027^∗∗∗^	−0.020^∗^
	(2.28)	(−2.19)	(2.75)	(−1.71)
fdi_3	−0.029	−0.013	0.019	0.040
	(−1.43)	(−1.07)	(0.58)	(0.89)
lnPGDP	0.093^∗^	0.296^∗∗^	0.237^∗∗^	0.329^∗∗∗^
	(1.69)	(2.10)	(2.28)	(3.85)
(lnPGDP)2	−0.102^∗^ (−1.90)	−0.166 (−0.95)	−0.261 (−1.25)	−0.193^∗^ (−1.76)
lnRd	−0.021	0.016	−0.010	−0.013^∗^
	(−1.59)	(0.78)	(−1.41)	(−1.74)
lnStr	−0.095^∗∗∗^	−0.093^∗∗∗^	−0.080^∗∗^	−0.084^∗∗^
	(−3.51)	(−3.64)	(−2.21)	(−2.26)
lnEdu	−0.032	−0.035	−0.029^∗^	−0.034^∗∗^
	(−1.14)	(−1.32)	(−1.77)	(−2.03)
Constant term	−0.373	0.049	0.503	−0.574^∗∗^
	(−1.57)	(1.31)	(0.94)	(−2.31)
*F* Value	252.36	287.09	171.74	190.53
	[0.000]	[0.000]	[0.000]	[0.000]
R2	0.65	0.67	0.53	0.55

## Data Availability

The data used to support the findings of this study can be obtained from the author upon request.

## References

[1] Rehmani S. S., Siddiqui S. H. (2019). Consumer’s attitude towards green supply chain practices and its impact on their intentions to buy at fast food restaurants in bahawalpur, Pakistan. *Sustainable Business and Society in Emerging Economies*.

[2] El-Kassar A. N., Singh S. K. (2019). Green innovation and organizational performance: the influence of big data and the moderating role of management commitment and HR practices. *Technological Forecasting and Social Change*.

[3] Pan X., Pan X., Song M., Guo R. (2019). The influence of green supply chain management on manufacturing enterprise performance: moderating effect of collaborative communication. *Production Planning & Control*.

[4] Zhao D. (2021). Choice of environmental and economic path for building a supply chain financial cloud ecosystem under the background of “internet +. *Wireless Communications and Mobile Computing*.

[5] Abdallah A. B., Al-Ghwayeen W. S. (2019). Green supply chain management and business performance: the mediating roles of environmental and operational performances. *Business Process Management Journal*.

[6] Lin Y. C., Zhang L. (2020). The impact of the greening tax system on sustainable development: a political economy perspective. *IOP Conference Series: Earth and Environmental Science*.

[7] Lin H. F. (2022). It resources and quality attributes: the impact on electronic green supply chain management implementation and performance. *Technology in Society*.

[8] Benuzh A., Mochalov I. (2020). Implementation of sustainable technology of green roofs for renovation in moscow. *IOP Conference Series: Materials Science And Engineering*.

[9] Mlt A., Msib C., Nk B., Faf B., Sa D. (2019). A literature review on green supply chain management: trends and future challenges - sciencedirect. Resources. *Conservation & Recycling*.

[10] Aslam H., Rashid K., Wahla A. R., Tahira U. (2018). Drivers of green supply chain management practices and their impact on firm performance: a developing country perspective. *Journal of Quantitative Methods*.

[11] Zhao F. (2021). The study of images in xu zhimo’s poetry of sayannala’s 18 poems and farewell to cambridge from the perspective of figure-ground theory in cognitive poetics. *Open Access Library Journal*.

[12] Ahmed W., Najmi A., Khan F. (2019). Examining the impact of institutional pressures and green supply chain management practices on firm performance. *Management of Environmental Quality: An International Journal*.

[13] Zhang X. W., Sui H. X., Sun K. Q., Mei-Jin L. I., Ding G. Y. (2019). Consideration of rural governance in chengdu from the perspective of the combination of autonomy, rule of law and rule of virtue in the new era. *Journal of University of Electronic Science and Technology of China*.

[14] Ghosh M. (2019). Determinants of green procurement implementation and its impact on firm performance. *Journal of Manufacturing Technology Management*.

[15] Liu Q. (2019). Research on usufructuary right and mining right from the perspective of green civil code. *Journal of Environmental Management College of China*.

[16] Khan M. T., Idrees M. D., Rauf M., Sami A., Ansari A., Jamil A. (2022). Green supply chain management practices’ impact on operational performance with the mediation of technological innovation. *Sustainability*.

[17] Wu W., Cheng Y., Lin X., Yao X. (2019). How does the implementation of the policy of electricity substitution influence green economic growth in China?. *Energy Policy*.

[18] Azimi H., Amiri V. (2018). Investigating the effect of market orientation on environmental performance with the mediating role of green supply chain management strategies case study khales sazan rooy company. *Journal of Advanced Research in Management*.

[19] Biao-Wen X. U., Wang H. P., Lin G. H. (2019). Application of policy instruments for green growth of agriculture in europe and America and its enlightenment. *Journal of Fujian Agriculture and Forestry University (Natural Science Edition)*.

[20] Yildiz Çankaya S., Sezen B. (2019). Effects of green supply chain management practices on sustainability performance. *Journal of Manufacturing Technology Management*.

[21] Fang C., Zhang J. (2018). Performance of green supply chain management: a systematic review and meta analysis. *Journal of Cleaner Production*.

[22] D’Amato D., Droste N., Winkler K. J., Toppinen A. (2019). Thinking green, circular or bio: eliciting researchers’ perspectives on a sustainable economy with q method. *Journal of Cleaner Production*.

[23] Sahoo S., Vijayvargy L. (2020). Green supply chain management practices and its impact on organizational performance: evidence from indian manufacturers. *Journal of Manufacturing Technology Management*.

[24] Lee C., Lim S., Ha B. (2021). Green supply chain management and its impact on consumer purchase decision as a marketing strategy: applying the theory of planned behavior. *Sustainability*.

[25] Wang X. Y., Guang-Pei L. I. (2018). A summary of research on green supply chain management, green design drivers and their impacts. *Logistics Engineering and Management*.

[26] Raj K. B., Srinivas K. (2019). Impact of robustness of supply chain on its performance - an empirical study. *Logistics Engineering and Management*.

[27] Acquaah M., Agyapong A., Aidoo S. (2021). Environmental orientation, green supply chain management, and institutional pressures on performance. *Academy of Management Proceedings*.

[28] Kitsis A. M., Chen I. J. (2021). Do stakeholder pressures influence green supply chain practices?exploring the mediating role of top management commitment. *Journal of Cleaner Production*.

